The article "ZASP Interacts with the Mechanosensing Protein Ankrd2 and p53 in the Signalling Network of Striated Muscle" was retracted in 2024. Reasons: duplicated images; overlap with earlier publications; original data or images not available; concerns about the images.

# ZASP Interacts with the Mechanosensing Protein Ankrd2 and p53 in the Signalling Network of Striated Muscle

**DOI:** 10.1371/journal.pone.0092259

**Published:** 2014-03-19

**Authors:** Valentina C. Martinelli, W. Buck Kyle, Snezana Kojic, Nicola Vitulo, Zhaohui Li, Anna Belgrano, Paolo Maiuri, Lawrence Banks, Matteo Vatta, Giorgio Valle, Georgine Faulkner

**Affiliations:** 1 International Centre for Genetic Engineering and Biotechnology, Trieste, Italy; 2 Department of Paediatrics (Cardiology), Baylor College of Medicine, Houston, Texas, United States of America; 3 Laboratory of Molecular Biology, Institute of Molecular Genetics and Genetic Engineering, University of Belgrade, Belgrade, Serbia; 4 Centro di Ricerca Interdipartimentale per le Biotecnologie Innovative, University of Padua, Padova, Italy; 5 Systems Cell Biology of Cell Polarity and Cell Division, Institut Curie, Paris, France; 6 Department of Medical and Molecular Genetics, University of Indiana, Indianapolis, Indiana, United States of America; Georgia Regents University, United States of America

## Abstract

ZASP is a cytoskeletal PDZ-LIM protein predominantly expressed in striated muscle. It forms multiprotein complexes and plays a pivotal role in the structural integrity of sarcomeres. Mutations in the ZASP protein are associated with myofibrillar myopathy, left ventricular non-compaction and dilated cardiomyopathy. The ablation of its murine homologue Cypher results in neonatal lethality. ZASP has several alternatively spliced isoforms, in this paper we clarify the nomenclature of its human isoforms as well as their dynamics and expression pattern in striated muscle. Interaction is demonstrated between ZASP and two new binding partners both of which have roles in signalling, regulation of gene expression and muscle differentiation; the mechanosensing protein Ankrd2 and the tumour suppressor protein p53. These proteins and ZASP form a triple complex that appears to facilitate poly-SUMOylation of p53. We also show the importance of two of its functional domains, the ZM-motif and the PDZ domain. The PDZ domain can bind directly to both Ankrd2 and p53 indicating that there is no competition between it and p53 for the same binding site on Ankrd2. However there is competition for this binding site between p53 and a region of the ZASP protein lacking the PDZ domain, but containing the ZM-motif. ZASP is negative regulator of p53 in transactivation experiments with the p53-responsive promoters, MDM2 and BAX. Mutations in the ZASP ZM-motif induce modification in protein turnover. In fact, two mutants, A165V and A171T, were not able to bind Ankrd2 and bound only poorly to alpha-actinin2. This is important since the A165V mutation is responsible for zaspopathy, a well characterized autosomal dominant distal myopathy. Although the mechanism by which this mutant causes disease is still unknown, this is the first indication of how a ZASP disease associated mutant protein differs from that of the wild type ZASP protein.

The article "ZASP Interacts with the Mechanosensing Protein Ankrd2 and p53 in the Signalling Network of Striated Muscle" was retracted in 2024. Reasons: duplicated images; overlap with earlier publications; original data or images not available; concerns about the images.

## Introduction

The Z-line acts as an interface between the contractile apparatus and the cytoskeleton connecting myofibrils to the sarcolemmal membrane, and hence the extracellular matrix. It is a focal point for sensing muscle activity and signal transduction that not only functions as a scaffold that links the contractile units by anchoring the actin and titin filaments of adjacent sarcomeres but also has a role in intra- and inter-cellular signalling pathways [1]. The Z-line is composed of a complex network of interacting proteins, with structural and/or regulatory functions that during muscle contraction transmit tension and force along the muscle fibre [2]. Proteins with a wide variety of functions bind to the Z-line, for example, proteins involved in ion channel interactions, cytoplasmic and nuclear signalling, enzymatic reactions and the cytoskeletal structure [3]. In the heart the Z-line anchors the ends of myofibrils in junctions known as intercalated discs that link the sarcomere laterally to the cell membrane via costameric proteins [4], [5]. In synthesis the Z-line is a node controlling contraction, intracellular signalling and striated muscle function as well as being a sensitive site whose disruption leads to myopathies [5], [6], [7], [8].

Z-band Alternative Spliced PDZ motif (ZASP) protein [9] is involved in maintenance of the Z-line and is highly expressed in striated muscle in both human [9] and mouse [10], [11], the murine homologue being termed Cypher [10]. The gene coding ZASP is also known as *LIM domain binding 3 (ldb3)* [12] and maps on chromosome 10q22.3-10q23.2. The ability of ZASP to maintain Z-band integrity during muscle contraction has been reported not only for mouse [13] but also for Zebrafish [14] and Drosophila [15], [16]. The number of ZASP exons, as well as the number of isoforms produced by alternative splicing, vary between species. For example, there are respectively sixteen and seventeen exons in human and mouse, giving rise to six isoforms reported so far for both species [9], [10], [17], [18].

ZASP is a member of the PDZ/LIM family [19], a class of Z-line proteins composed of two sub-families, the ALP and Enigma. In addition to a PDZ domain, mammalian members have either one LIM domain (ALP) or 3 LIM domains (Enigma). The PDZ domain mediates protein-protein interactions by normally binding to the extreme C-terminal amino acids (last 4 to 6 aa) of its binding partners [20]. LIM domains have eight conserved cysteine and histidine residues that form a motif composed of two tandemly repeated zinc fingers [21]. Functionally, LIM domains mediate protein-protein interactions and have diverse cellular roles such as regulators of gene expression, cell adhesion, cell motility and signal transduction. ZASP belongs to the Enigma sub-family and has isoforms with one PDZ domain and either none or three LIM domains [9], [10], [11], whereas in Drosophila Zasp52 has one PDZ domain and six LIM domains [15], [22] and Drosophila Zasp66 has one PDZ domain and another domain [15], [23] with some similarity to the short 26 amino acid region, known as the ZASP-like Motif (ZM) found in some members of the ALP (ALP, CLP-36) and Enigma (ZASP) sub-families of proteins [24], [25].

The article "ZASP Interacts with the Mechanosensing Protein Ankrd2 and p53 in the Signalling Network of Striated Muscle" was retracted in 2024. Reasons: duplicated images; overlap with earlier publications; original data or images not available; concerns about the images.

In mammalian isoforms of ZASP, the ZM is encoded either by exon 4 or 6 [24], or in some cases both. Alpha-actinin2 binds ZASP via both the ZM region and the PDZ domain [24], [26]. The PDZ region of ZASP not only interacts with alpha-actinin2 [9], [10] but also with proteins of the FATZ/calsarcin/myozenin family [27], [28] and the Myotilin (myotilin, myopalladin, palladin) family [28]. Recently in studies using human embryonic kidney-293 cells and neonatal rat cardiomyocytes, the PDZ domain of ZASP was found to bind telethonin (T-Cap) forming a complex with the sodium channel Na(v)1.5 [29]. ZASP has also been reported to bind nebulette [30], and phosphoglucomutase 1 [31]. Interestingly phosphoglucomutase1 binds to the ZM-motif of ZASP and also to a region encoded by exon 10 [31].

Point mutations in the human *ldb3 (ZASP)* gene have been identified in patients with various myopathies such as dilated cardiomyopathy (DCM) [17], [32], left ventricular non-compaction (LVNC) [17], [32], hypertrophic cardiomyopathy [33] and inclusion body myositis [34] as well as in patients with an autosomal dominant form of progressive muscular dystrophy termed zaspopathy [35], [36]. Zaspopathy is one of a collection of myofibrillar myopathies (MFMs) caused by mutations in a variety of Z-line proteins, however mutations in ZASP cause the highest percentage of MFM cases [37].

Most of the disease associated mutations in *ZASP* are located in exons 4 and 6, known to code for the ZM-motif [17], [35], [36]. To investigate whether these mutations could perturb the normal dynamic properties of ZASP, the mobility of the various ZASP isoforms and mutants was measured using fluorescence recovery after photobleaching (FRAP) [38] and marked differences were detected.

Many sarcomeric proteins, including ZASP, have been reported to have multiple binding partners [28], [39], [40]. Previously, we had shown that RIL and hCLIM proteins, two members of the ALP/Engima family, were able to interact with the mechanosensing protein Ankrd2 via their PDZ domain [41], therefore it was possible that ZASP could also interact with Ankrd2. Ankrd2 is an ankyrin repeat protein, mainly expressed in striated muscle [42], in the sarcomeric I-line, adjacent to the Z-line [43], [44]. Its location is affected by differentiation, being located mainly in the nucleus in myoblasts and the cytoplasm in myotubes [42], [45].

The article "ZASP Interacts with the Mechanosensing Protein Ankrd2 and p53 in the Signalling Network of Striated Muscle" was retracted in 2024. Reasons: duplicated images; overlap with earlier publications; original data or images not available; concerns about the images.

Here, we confirm our hypothesis that ZASP binds Ankrd2. Moreover, we were able to show that two ZASP mutants with mutations in the ZM-motif region were unable to bind Ankrd2 and could only bind weakly to alpha-actinin2. We also discovered another new binding partner for ZASP, the nuclear phosphoprotein p53, that is also known to bind Ankrd2 [42] and telethonin [46]. Both Ankrd2 and p53 are involved in signalling, regulation of gene expression and muscle differentiation [41]. ZASP, Ankrd2 and p53 were found to form a trimeric complex, with the functional consequence of decreased activity of the p53-responsive promoters, BAX and MDM2 in transactivation experiments.

## Results

### Nomenclature of Human ZASP Isoforms

The results presented in this paper pertain to human isoforms of cardiac and skeletal muscle, therefore the name ZASP will be used throughout the paper. However when discussing data from the literature pertaining to mouse isoforms the name Cypher will be used [10]. Multiple alternatively spliced isoforms of the ZASP protein are coded by the human *ldb3* gene that has 16 exons in human and 17 exons in mouse [17], [18]. There are several discrepancies in the nomenclature of human ZASP isoforms, the numbering differing from the original literature and also between databases.

In this paper we use the nomenclature of the UniProtKB human database (www.uniprot.org) with the difference that the ldb3 isoforms 1–7 will be designated as ZASP1–ZASP7 (Table 1). We detected a new human isoform named ZASP8, which contains exons 1–4, 7, 8 and 11–16 (Table 1), as established by sequence analysis of the PCR products and multiple primer combinations. Its transcript was deposited in the Genbank database as LDB3-8 KF772970 [47]. A similar sequence had already been deposited in GenBank as AK294696 [48], that encodes a protein named BAG57855.1 (or B4DGP4 in UniProtKB/TrEMBL). Although the genomic sequence for exon 12 is the same for both transcripts, AK294696 differs from ZASP8 in that it has an odd splicing pattern for exon 12 in which the first 63 bp are present, then 48 bp are spliced out or not transcribed, and the sequence restarts again at base 112. Since no donor/acceptor sites are present we have no explanation for this. To further clarify the isoforms of ZASP a supplementary table (Table S1) has been included listing the Cypher isoforms found in mouse and their tissue specificity. The comparison of the Cypher and ZASP isoforms was done using BLASTP and the most similar (highest percentage identity) were listed in Table S1.

The article "ZASP Interacts with the Mechanosensing Protein Ankrd2 and p53 in the Signalling Network of Striated Muscle" was retracted in 2024. Reasons: duplicated images; overlap with earlier publications; original data or images not available; concerns about the images.

**Table 1:** Nomenclature of human ZASP isoforms.

LDB3/ZASP UniProtKB	ZASP Isoforms	Protein (aa)	Motifs^**^	GenBank transcripts	ENSEMBL-LDB3 transcript	Exons
**ZASP1** O75112-1	C/Z4^*^	727	ZM4 LIM	LDB3 var 1 NM_007078.2	LDB3-001 ENST00000361373	1, 2, 3, 4, 7, 8, 10, 11, 12, 13, 14, 15, 16
**ZASP2** O75112-2	ZASP v3^#^ C/Z3*	617	ZM6 LIM	LDB3 var 2 NM_001080114.1	LDB3-201 ENST00000263066	1, 2, 3, 5, 6, 7, 8, 11, 12, 13, 14, 15, 16
**ZASP3** O75112-3	ZASP v2^#^ C/Z2^*^	470	LIM	ZASP var 2 AJ133768.1	LDB3-203 ENST00000352360	1, 2, 3, 11, 12, 13, 14, 15, 16
**ZASP4** O75112-4	C/Z6^*^	398	ZM4 ZM6	LDB3 var 6 NM_001171611.1	LDB3-204 ENST00000372056	1, 2, 3, 4, 6, 7, 8, 9
**ZASP5** O75112-5	ZASP-4^§^	330	ZM4	LDB3 var 3 NM_001080115.1	LDB3-202 ENST00000310944	1, 2, 3, 4, 7, 8, 9
**ZASP6** O75112-6	ZASP1^#^ C/Z1^*^	283	ZM6	LDB3 var 4 NM_001080116.1	LDB3-002 ENST00000372066	1, 2, 3, 5, 6, 7, 8, 9
**ZASP7** O75112-7	C/Z5^*^	732	ZM4 ZM6LIM	LDB3 var 5 NM_001171610.1	LDB3-205 ENST00000429277	1, 2, 3, 4, 6, 7, 8, 11, 12, 13, 14, 15, 16
**ZASP8**	ZASP8^¤^	664	ZM4 LIM	LDB3-var 8 KF772970	N/A	1, 2, 3, 4,7, 8, 11, 12, 13, 14, 15, 16

N/A not applicable. Original references for the ZASP isoforms are [# 9, *17 ¤47, §93]. **All ZASP isoforms have a PDZ domain.

### The Expression Pattern of Human ZASP Isoforms

Initially we used quantitative (real-time) polymerase chain reaction (qPCR) to determine the level of expression of individual isoforms of ZASP in adult human striated muscle compared to GAPDH used as a reference gene (Figure S1). Limitation in amplicon size and the similarity between isoforms rendered impossible quantification of each individual isoform using qPCR. Therefore the isoforms were sorted into three groups according to similarity in the exon coding for the ZM-motif. As seen in Figure S1, Group 1 and Group 2 isoforms were expressed in both human adult cardiac and skeletal RNA, Group 1 being the most highly expressed. The isoforms in Group 3 were only detectable in heart not in skeletal muscle. To clarify the expression pattern of the individual ZASP isoforms, RNAseq was performed using mRNA from both human adult and foetal skeletal and cardiac muscle tissue (Table 2). RNAseq can provide transcript level resolution of gene expression, however mapping fragments to isoforms is not a straightforward task. The Cufflinks program [49] was integrated with the process of mapping reads directly to the splice sites of ZASP isoforms in order to analyse the RNAseq data. The splicing site coverage analysis was performed for each transcript as detailed in the Materials and Methods, an isoform was considered to be expressed only if all of its splicing sites were confirmed (Table S2). The results of the RNAseq analysis for the human ZASP isoforms are summarised in Table 2 and given in detail including Cufflinks data in Table S3. To render the tag counts (the number of sequenced reads that align to a gene of interest) comparable among the samples, a normalization was performed by the RPKM (reads per kilobase per million) method, widely used in RNAseq analysis (Table S3). The cut-off value is the number of reads mapped for every splice site in the isoforms and allows an estimate of the level of expression of the isoforms present in cardiac and skeletal muscle. Empirically the higher the cut-off, the higher is the level of expression of the isoform. Here we used cut-off values of 5, 2 and 1, meaning that at least 5, 2 or 1 reads were confirmed for each splicing site per isoform. Only ZASP3 was unable to be detected and that together with its peculiar splice pattern raises the question as to whether this isoform exists.

The article "ZASP Interacts with the Mechanosensing Protein Ankrd2 and p53 in the Signalling Network of Striated Muscle" was retracted in 2024. Reasons: duplicated images; overlap with earlier publications; original data or images not available; concerns about the images.

**Table 2:** Expression levels of human ZASP isoforms in striated muscle estimated from RNAseq data.

ZASP/LDB3	Adult heart	Foetal heart	Adult skeletal muscle	Foetal skeletal muscle
**ZASP1**	++	+++	+	++
**ZASP2**	+++	−	+++	+++
**ZASP3**	−	−	−	−
**ZASP4**	−	−	+	−
**ZASP5**	+++	+++	+	++
**ZASP6**	+++	−	+++	+++
**ZASP7**	−	−	+	−
**ZASP8**	+++	+++	+	++

The presence of each isoform is estimated on the bases of the number of reads mapping over the splice sites of the transcripts, respectively, 1, 2 and 5 reads (+, ++, +++) that give an indication of the level of expression determined by the coverage of each splice site of the transcript.

The data obtained by RNAseq (Table 2) is similar to that from qPCR (Figure S1), however in Group 1 it is likely that only ZASP isoforms 2 and 6 contributed to the qPCR value as we cannot detect ZASP3. Both by qPCR and RNAseq ZASP2 and ZASP6 are the most highly expressed isoforms in adult striated muscle while ZASP1, ZASP5 and ZASP 8 (Group 2) are more highly expressed in cardiac than in skeletal muscle. In contrast to the qPCR data, the RNAseq data shows that ZASP4 and ZASP7 (Group 3) are poorly expressed in adult skeletal muscle and not expressed in heart (Table 2). In foetal tissue ZASP1, ZASP5 and ZASP8, that have exon 4, are expressed in both heart and skeletal muscle although more highly in heart whereas ZASP2 and ZASP6, that have exon 6, are highly expressed in skeletal muscle but not in heart. ZASP4 and ZASP7 are not detected in either heart or skeletal foetal muscle.

The article "ZASP Interacts with the Mechanosensing Protein Ankrd2 and p53 in the Signalling Network of Striated Muscle" was retracted in 2024. Reasons: duplicated images; overlap with earlier publications; original data or images not available; concerns about the images.

### Intracellular Localization of ZASP Isoforms

To determine the intracellular localization of some of the ZASP isoforms, standard epifluorescence microscopy was performed on murine skeletal myoblasts C2C12 transfected with plasmids expressing recombinant ZASP1, 5, 6 and 8 fused with GFP protein. Tagged recombinant proteins were used in order to discriminate between the endogenous Cypher and human ZASP protein. Of the isoforms chosen both ZASP5 and ZASP6 are short isoforms without LIM domains, their ZM-motif being coded by exon 4 and 6, respectively. ZASP1 and ZASP8 are long isoforms with LIM domains, their ZM-motif being coded by exon 4. In transfected C2C12 cells all four isoforms localized in a similar pattern along the actin stress fibres (Figure S2A) that were stained with rhodamine-phalloidin. Apart from actin, ZASP6 is known to co-localise with alpha-actinin2 [9], [10] therefore in order to determine if the other ZASP isoforms studied showed the same pattern of co-localisation, transfected C2C12 cells were probed with monoclonal anti-alpha-actinin2 antibody. As expected, co-localisation was seen for alpha-actinin2 and the tested ZASP isoforms (Figure S2B).

### Comparison of the Dynamics of Human ZASP Isoforms

Since no major differences in intracellular localization could be detected between the ZASP isoforms 1, 5, 6 and 8, we used FRAP to compare the dynamics of the different isoforms. Analysis of fluorescence recovery can be used to determine the kinetic parameters of a protein, including its diffusion constant, mobile fraction, transport rate or binding/dissociation rates [50]. Moreover, FRAP measures the ability of the isoforms to form stable protein complexes, in fact, Wang and colleagues used this method to study the dynamics of the Z-band proteins such as Cypher1 s and 2 s, telethonin, alpha-actinin2, myotilin and actin in skeletal muscle cells [51]. It should be emphasised that actively growing murine myoblasts (C2C12) are mono-nucleated cells that have non-orientated actin filaments and behave like activated skeletal muscle satellite cells [52], and at this stage they do not have either premyofibril Z-bodies or Z-lines.

C2C12 were transfected with vectors expressing GFP-ZASP isoforms. To determine their fluorescence recovery rates, the fluorescence intensity data for each trial were normalized [53] and the fluorescence recovery was plotted as a function of time after bleaching. The FRAP data were fitted with a reaction-diffusion model [54] to extract the mobile fraction (MF%) and recovery rate constants. The rates of fluorescence recovery for the isoforms were markedly different as can be seen from the FRAP results plotted in Figure 1A and given in detail in Tables S4 and S5. The four ZASP isoforms had different MF% values: 100% for ZASP5, 98% for ZASP1, 92% for ZASP8 and 70% for ZASP6 of the initial intensity within 10 min. ZASP1 and ZASP5 recover faster than either ZASP6 or ZASP8, as shown in Figure S3.

The article "ZASP Interacts with the Mechanosensing Protein Ankrd2 and p53 in the Signalling Network of Striated Muscle" was retracted in 2024. Reasons: duplicated images; overlap with earlier publications; original data or images not available; concerns about the images.

**Figure 1:** FRAP analysis of human isoforms of ZASP and their mutants. The recovery times were measured every 10–12 sec, within 10 min after bleaching (50 points). The relative FRAP recovery was plotted as a function of time. **A)** FRAP analysis of ZASP isoforms, 1 (black squares), 5 (white diamonds), 6 (black circles) and 8 (white triangles). **B)** FRAP analysis of human ZASP6 (black circles) and its mutants ZASP6_K136M (white diamonds), ZASP6_D117N (white squares), ZASP6_A171T (white cross), ZASP-6_A147T (white saltire cross), ZASP6_A165V (white circles). **C)** FRAP analysis comparing the ZASP1 wt (black square) and ZASP1 mutant S189L (white circles).

When the FRAP profiles of the isoforms are compared (Figure 1A) the most dynamic is ZASP5 (35.6 kDa) and the least ZASP6 (31 kDa) which is very interesting as both proteins have similar molecular weights (MWs), the main difference being their ZM-motifs, encoded respectively by exon 4 and exon 6. In contrast, ZASP1 (77 kDa) and ZASP5 (35.6 kDa) are both fully mobile although they have different MWs but the same ZM-motif encoded by exon 4 (Figure 1A). ZASP1 (77 kDa) and ZASP8 (71.3 kDa) have similar MWs and the same ZM-motif encoded by exon 4, however they showed differences in fluorescence recovery. ZASP8 recovered at a slower rate than ZASP1 (Figure 1A, Figure S3) but had a similar diffusion coefficient and a better binding affinity (Table S4). The ZASP6 isoform had a much slower recovery rate and an higher immobile fraction compared to the other isoforms, indicating a better binding capacity (Table S4). Therefore once ZASP6 binds, its binding is maintained longer, the possible consequence is stronger and more efficient binding when compared with the other isoforms. Since the recovery kinetics reflects the mobility of the protein, these data suggest that the recovery of the ZASP isoforms is mainly affected by their binding capacity rather than by their diffusion coefficient. Indeed ZASP1 recovers significantly faster than ZASP6 even although it has a higher mass and a lower diffusion coefficient. It is evident that the differences in the extent of recovery were not due to the presence/absence of the three LIM domains but may be due to differences in the ZM-motif. ZASP6 is the only isoform with its ZM-motif encoded by exon 6, and it has the slowest recovery, therefore it is reasonable to suggest that the ability to undergo a binding event, as well as its specificity and duration could be due to the ZM-motif.

The article "ZASP Interacts with the Mechanosensing Protein Ankrd2 and p53 in the Signalling Network of Striated Muscle" was retracted in 2024. Reasons: duplicated images; overlap with earlier publications; original data or images not available; concerns about the images.

### Comparison of the Dynamics of Isoforms ZASP1 and ZASP6 and their Mutants

The majority of ZASP point-mutations, associated with disease, are located in exons 4 and 6. As different isoforms have variable dynamic properties it was important to compare mutations with their non-mutated counterpart. We tested zaspopathy associated ZASP6 isoforms with mutations in its ZM-motif in exon 6: pA147T and pA165V [35]. Mutants outside of the ZM-motif are ZASP6_D117N (in exon 6) detected in LVNC and conduction disturbances [17], [29], ZASP6_A171T (Anna Belgrano, unpublished) and ZASP6_K136M associated with DCM [17].

Disease associated specific point mutations were introduced by site-directed mutagenesis into ZASP cDNA, cloned in GFP expression vectors and transfected into C2C12 cells. FRAP experiments were performed to investigate whether these mutations could perturb the normal dynamic properties of ZASP. The results show that the mutants of ZASP6 had markedly different dynamics compared to ZASP6 wt (Figure 1B, Tables S4 and S5), having significantly higher recovery rates after 10 min compared to the wt. Although the mutants have similar mass and share similar diffusion coefficients (Coeff-Diff) with the wild type ZASP6, the specificity of binding strongly decreases (K<<1), indeed the mutants bind for a shorter time and with lower efficiency when compared to ZASP6 wt (Table S4). The decrease in binding specificity appears to be associated with the site of localization of the point mutation in the protein. Mutants that have a point mutation in the ZM-motif (aa 148–173) or very close to it show a higher decrease in binding efficiency. ZASP6_A165V, with a mutation in the middle of the ZM-motif, has the highest recovery rate, 99% in 10 min, indicating a very low binding efficiency, similar to that of ZASP1 wt (98%) (Table S4). This mutation has a profound effect on the mobility of the protein within the cell and it is probably not coincidental that it is the best studied in MFM.

ZASP1 has its ZM-motif (aa 189–214) encoded by exon 4. Mutant ZASP1_S189L [17], associated with LVCN [55], was originally designated ZASP1_S196L, as the original ZASP transcript had an additional 21 bp currently not considered in new annotations. The ZASP1_S189L (Figure 1C, Table S5) has a slower recovery rate and a lower MF% (89%) compared to ZASP1 wt (98%). Thus it is interesting to note that this particular mutation of ZASP1 seems to increase the specificity of its binding. From the results of the FRAP experiments it would appear that the ZM-motif is important since alterations in this region can drastically alter the dynamic properties of the ZASP proteins.

The article "ZASP Interacts with the Mechanosensing Protein Ankrd2 and p53 in the Signalling Network of Striated Muscle" was retracted in 2024. Reasons: duplicated images; overlap with earlier publications; original data or images not available; concerns about the images.

### ZASP6 Interacts with Ankrd2

Previously we had shown that Ankrd2 was able to interact with some PDZ-LIM proteins via their PDZ domain [41]. Since ZASP6 is also a member of this family, it was possible that it could bind Ankrd2. To test this hypothesis co-immunoprecipitation (Co-IP) experiments were performed with cell lysates of transfected COS-7, immunoprecipitated with anti-FLAG antibody and probed with anti-Ankrd2 antibody. Figure 2A shows that FLAG-ZASP6 was able to interact with cMyc-Ankrd2. No non-specific interactions were observed. However since ZASP6 can bind proteins via its PDZ and/or ZM-motif it was important to investigate which domain could function as interaction site for Ankrd2.

**Figure 2:** PDZ and ZM1 regions of ZASP6 directly bind Ankrd2. **A)** Co-IP of ZASP6 and Ankrd2 using lysates of COS-7 cells transfected with the indicated combination of pCMV vectors expressing cMyc-Ankrd2 and FLAG-ZASP6. Immunoprecipitation was performed with anti-FLAG antibody. The presence of Ankrd2 in the immune complex was confirmed by probing the membrane with mouse polyclonal anti-Ankrd2 antibody (upper panel). As controls, the cell lysates were tested with polyclonal antibodies to anti-Ankrd2 (middle panel) and anti-ZASP6 (bottom panel). **B)** Co-IP of PDZ-ZASP6 and Ankrd2 using lysates of COS-7 cells transfected with cMyc-Ankrd2 and pEGFP-PDZ as indicated. The cell lysates were immunoprecipitated with an anti-cMyc monoclonal antibody and probed with a polyclonal goat anti-GFP antibody conjugated to HRP (upper panel). Comparable expression levels of Ankrd2 and PDZ-ZASP6, weredemonstrated by probing the membrane with a mouse anti-Ankrd2 polyclonal antibody (middle panel) and rabbit anti-GFP polyclonal antibody (lower panel). **C)** Co-IP of ZM1-ZASP6 and Ankrd2 using lysates of COS-7 cells transfected with cMyc-Ankrd2 and FLAG-ZM1 as indicated. Ankrd2 was immunoprecipitated with anti-FLAG EZview resin and detected with an anti-Ankrd2 mouse polyclonal antibody (upper panel). As controls, cell lysates were tested with an anti-Ankrd2 mouse polyclonal antibody (middle panel) and with an anti-FLAG rabbit polyclonal antibody (bottom panel). All secondary antibodies were conjugated with HRP. **D)** GST-overlay assay with purified recombinant proteins expressed in *E. coli*. His-Ankrd2 (4 μg) was separated by SDS-PAGE, blotted and membrane strips were incubated with 4 μg of either GST-ZASP6, GST-PDZ, GST-ZM1 or GST alone, washed and then probed with anti-GST goat polyclonal antibody. As a control, an anti-histidine antibody was used to probe membrane strips identical to those used for the overlay to show that the His-Ankrd2 protein was equally loaded (lower panel). **E)** A schematic diagram of ZASP6 showing the positions of the PDZ domain (aa 11–84) and ZM-motif (aa 148–173). In this study the expression vectors with constructs for PDZ and ZM1 (ZASP6 without the PDZ domain) expressed respectively 85 and 197 amino acid fragments of ZASP6.

The article "ZASP Interacts with the Mechanosensing Protein Ankrd2 and p53 in the Signalling Network of Striated Muscle" was retracted in 2024. Reasons: duplicated images; overlap with earlier publications; original data or images not available; concerns about the images.

In order to do this the PDZ and ZM1 (ZASP6 without the PDZ domain) regions of ZASP6 were cloned into a GFP expression vector and used in Co-IP experiments. COS-7 cells were transfected with vectors expressing cMyc-Ankrd2 and GFP-PDZ (Figure 2B) or FLAG-ZM1 (Figure 2C). Recombinant proteins were immunoprecipitated with anti c-Myc mouse monoclonal antibody and probed with anti-GFP rabbit polyclonal antibody (Figure 2B). A positive band (second column) was detected in the double transfection indicating that the PDZ domain of ZASP6 is sufficient to interact with Ankrd2. No cross-reactions were detected (third and fourth columns).

In Figure 2C the lysates were immunoprecipitated using anti-FLAG antibody and Ankrd2 was detected with anti-Ankrd2 polyclonal antibody. A strong positive band was detected in the double transfection, indicating that the ZASP6 without the PDZ domain (ZM1) is also able to bind Ankrd2 (second column). No cross reactions were detected (third and fourth columns). Therefore Ankrd2 can bind ZASP6 via its PDZ domain alone (Figure 2B) and/or via the domains present in ZM1 region, most probably ZM-motif (Figure 2C).

Since the binding between ZASP6 and Ankrd2 was detected using cell lysates, the presence of an intermediary protein involved in the binding could not be ruled out. Therefore a GST-overlay experiment was performed (Figure 2D). Immunoblotted purified His-Ankrd2 protein was incubated with either GST-ZASP6, GST-PDZ, GST-ZM or GST alone, then probed with anti-GST antibody. His-Ankrd2 protein was equally loaded in each lane (Figure 2D, lower panel). The results of the GST-overlay assay demonstrate that the His-Ankrd2 protein bound the GST-ZASP6, GST-PDZ and GST-ZM1 proteins, although the latter binding appears to be weaker. No interactions were detected with either the GST alone or with the His-Ankrd2 protein alone thus excluding any possible non-specific interactions. The interaction between ZASP6 and Ankrd2 would appear to be direct as no other intermediary proteins were present in the overlay assay. In Figure 2E is a schematic diagram showing the positions of the PDZ (11–84 aa) and ZM (148–173 aa) domains in the ZASP6 protein (SMART program, EMBL).

The article "ZASP Interacts with the Mechanosensing Protein Ankrd2 and p53 in the Signalling Network of Striated Muscle" was retracted in 2024. Reasons: duplicated images; overlap with earlier publications; original data or images not available; concerns about the images.

In conclusion the ZASP6 protein can bind directly to the Ankrd2 protein via both its PDZ domain and its ZM1 region, which includes the ZM-motif and the C-terminus of the protein.

### The ZASP6 Binding Site is Located in the Ankyrin Repeat Region of Ankrd2

The Ankrd2 used in this paper corresponds to human Ankrd2-001 (ENST00000370655) a transcript encoding a 333 aa protein however the designated canonical Ankrd2 is now Ankrd2-202 (ENST00000307518) a transcript that encodes a 360 aa protein. This difference is due to the existence of alternative initiation sites for human Ankrd2. Figure 3A shows a schematic diagram of the different regions of Ankrd2 used in this experiment, the numbering refers to the canonical Ankrd2-202 sequence, FL was full-length for Ankrd2-001 [42] missing the first 32 aa of the canonical Ankrd2. The deletants of the Ankrd2 protein used were the following: N-terminus (N, aa 32–147); N terminus with ankyrin repeats (NA, aa 32–311); C terminus with ankyrin repeats (CA, aa 148–360) and C-terminus (C, aa 306–360).

**Figure 3:** ZASP6 interacts with the ankyrin repeat region of Ankrd2. **A)** is a schematic diagram showing the different regions of Ankrd2 used in this experiment. The Ankrd2 numbering refers to the canonical Ankrd2-202 sequence (ENSEMBL); FL refers to the full-length of Ankrd2-001 (Kojic et al., 2004). There are four ankyrin repeat motifs in the human Ankrd2 protein between aa 148–308, a PEST sequence that targets proteins for proteolytic cleavage, as well as regions rich in amino acids lysine (K) and proline (P). **B)** GST-overlay assay demonstrating that NA and CA regions of Ankrd2 contain the binding site/sites for ZASP6. GST-FL-Ankrd2, GST-N-Ankrd2, GST-NA-Ankrd2, GST-CA- Ankrd2, GST-C-Ankrd2 and GST alone were separated by SDS-PAGE and blotted. The membrane was blocked and then overlaid with lysate from COS-7 cells transfected with pcDNA3-HA-ZASP6. The membrane was probed with an anti-ZASP mouse polyclonal antibody. The Western blot in the lower panel shows that equal amounts of the GST proteins were used in this experiment.

In order to map ZASP6 binding sites on Ankrd2, an overlay assay was performed (Figure 3B). Ankrd2 deletants, expressed as recombinant GST proteins, were separated by SDS-PAGE and blotted. The membrane was overlaid with lysate from COS-7 cells transfected with HA-ZASP6 and probed with a ZASP polyclonal antibody. Binding was detected between ZASP6 and GST-FL-Ankrd2, GST-NA-Ankrd2 and GST-CA-Ankrd2. The Western blot in the lower panel shows that equal amounts of the GST proteins were used in this experiment. From this result the binding site for ZASP6 would appear to be in the Ankyrin repeat region (aa 148–306) since HA-ZASP6 was found to interact with NA-and CA-regions of Ankrd2, but not with N- and C-terminal fragments.

The article "ZASP Interacts with the Mechanosensing Protein Ankrd2 and p53 in the Signalling Network of Striated Muscle" was retracted in 2024. Reasons: duplicated images; overlap with earlier publications; original data or images not available; concerns about the images.

### Interaction of ZASP6 Mutants with Alpha-actinin2 and Ankrd2

ZASP can bind alpha-actinin2 via both its PDZ [9], [10], [26] and its ZM [24], [25] domains. In fact, mutations in the PDZ domain of Cypher are known to alter its binding to alpha-actinin2 [55]. Are mutations in another binding site, namely the ZM-like motif, able to perturb interaction between ZASP and its binding partners? The results of the FRAP experiments showed dynamic differences between wt ZASP6 and its mutants that could be the result of disruption of the binding between these mutants and an unknown binding protein of ZASP. As these mutations are in the ZM-motif binding site the most likely interaction to be disrupted would be that of ZASP and alpha-actinin2.

In order to confirm this assumption Co-IP experiments were performed using COS-7 cells expressing cMyc-alpha-actinin2 and FLAG-ZASP6 wt protein or different mutants: ZASP6_K136M, ZASP6_A147T, ZASP6_A165V and ZASP6_A171T as well (Figure 4A). Cell lysates were immunoprecipitated with an anti-FLAG antibody and then subjected to SDS-PAGE, blotted and probed with an alpha-actinin2 antibody (Figure 4A). Alpha-actinin2 was able to bind mutants GFP-ZASP6_K136M and GFP-ZASP6_A147T, as efficiently as the wt ZASP6. Interestingly, the pA165V and pA171T mutations in the ZM-motif significantly reduced the ability of ZASP6 to interact with alpha-actinin2, demonstrating that the interaction between them is dependent on the integrity of ZM-motif. However, using confocal microscopy we did not see any difference in the co-localization of alpha-actinin2, with the ZASP6 mutants, compared to ZASP6 wt or with the ZASP1_S189L compared to the wt ZASP1 (data not shown) confirming previous findings [17].

**Figure 4:** Mutations in ZASP6 affect its interaction with alpha-actinin2 and Ankrd2. Wt and mutants of the ZASP6 isoform fused with FLAG (**A**) or GFP (**B**) tag were co-expressed with cMyc-alpha-actinin2 (**A**) or cMyc-Ankrd2 (**B**) in COS-7 cells as indicated. Protein extracts were immunoprecipitated with polyclonal antibodies to FLAG (**A**) or cMyc (**B**) tag. Precipitated proteins were analyzed by SDS-PAGE followed by Western blotting using rabbit anti-alpha actinin2 (**A**) or mouse anti-ZASP antibody (**B**). As controls, the lysates were probed with polyclonal antibodies to ZASP (**A** and **B**, middle panels), alpha-actinin2 (**A**, bottom panel) and mouse anti-Ankrd2 (**B**, bottom panel). The arrows in A and B, middle panels, show the major ZASP6 band.

The article "ZASP Interacts with the Mechanosensing Protein Ankrd2 and p53 in the Signalling Network of Striated Muscle" was retracted in 2024. Reasons: duplicated images; overlap with earlier publications; original data or images not available; concerns about the images.

The ZM-motif of ZASP6 not only binds alpha-actinin2 but also Ankrd2, therefore it is possible that the point mutations in the ZM-motif will alter the interaction between Ankrd2 and ZASP6. To test this hypothesis a Co-IP experiment was performed (Figure 4B). GFP-ZASP6 wt and different GFP-ZASP6 mutants: pK136M, pA147T, pA165V and pA171T were expressed in COS-7 cells in conjunction with cMyc-Ankrd2. Cell lysates were immunoprecipitated with an anti-cMyc antibody, subjected to SDS-PAGE, blotted and then probed with a ZASP antibody. Ankrd2 could bind the ZASP6_K136M and ZASP6_A147T mutants as well as ZASP6 wt but not the mutants in the ZM-motif ZASP_A165V and ZASP6_A171T (Figure 4B). In fact these mutants are completely defective in binding Ankrd2 whereas they still showed some binding to alpha-actinin2.

### ZASP6 Interacts with p53

We had previously shown that Ankrd2 can interact with p53 [42] and here we demonstrated that ZASP can bind Ankrd2, therefore we hypothesized that p53 may affect the binding of Ankrd2 to ZASP either by sequestering Ankrd2 or by forming a complex with ZASP and Ankrd2. Can p53 bind ZASP? This possibility was verified in a series of experiments, including Co-IP. In order to avoid interference from endogenous p53, the experiments were performed in p53^−/−^ H1299 cells. These cells were transfected with vectors expressing GFP-ZASP6, GFP-PDZ and p53 (Figure 5A). Cell lysates were immunoprecipitated with anti-p53 antibody and ZASP6 was visualized with anti-GFP antibody. As controls, cell lysates were blotted and probed with anti-GFP and anti-p53 antibodies. Non-specific interactions were not detected. The bands seen indicated that binding occurred between p53 and the ZASP6-PDZ domain as well as the full-length ZASP6 (Figure 5A). Therefore p53 is able to bind not only full-length ZASP6 but also its PDZ domain. Can the ZASP6 protein without the PDZ domain (ZM1) bind p53? H1299 cells were transfected with vectors expressing FLAG-ZASP6, FLAG-ZM1 and p53. Transfected cell lysates were immunoprecipitated with an anti-FLAG antibody. The proteins were separated by SDS-PAGE, blotted and probed with anti-p53 antibody. As controls, cell lysates were blotted and probed with anti-FLAG and anti-p53 antibodies, there were no cross reactions. A positive band was detected in the double transfections indicating that the ZASP6-ZM1 region as well as ZASP6 full-length bound to p53 (Figure 5B).

**Figure 5:** Binding between the PDZ domain of ZASP6 and p53 is direct, while interaction of p53 with ZM1 requires mediation of another protein/proteins. H1299 cells lacking endogenous p53,were transfected with pcDNA3-p53, GFP-ZASP6, GFP-PDZ and FLAG-ZM1, as indicated. Transfected cell lysates were incubated with (**A**) anti-p53 monoclonal antibody or (**B**) with anti-FLAG antibody immobilized on resin. Precipitated immune complexes were separated by SDS-PAGE. Immunoblotting was performed with anti-GFP polyclonal antibody (**A**, top panel) or anti-p53 (**B**, top panel). As controls, cell lysates were probed with rabbit polyclonal anti-GFP antibody (**A**, middle panel), monoclonal antibody to FLAG (**B,** middle panel) and anti-p53 monoclonal antibody (**A** and **B**, bottom panels). **C)** GST-overlay assay with purified His-p53 (4 μg), separated by SDS PAGE, transferred to Immobilon P membrane and overlaid with GST-ZASP6, GST-PDZ, GST-ZM1 or GST alone. GST proteins bound to p53 was detected by anti-GST polyclonal antibody. In the bottom panel, an identical membrane was probed with an anti-Histidine antibody to demonstrate that the same amount of His-p53 protein was loaded.

The article "ZASP Interacts with the Mechanosensing Protein Ankrd2 and p53 in the Signalling Network of Striated Muscle" was retracted in 2024. Reasons: duplicated images; overlap with earlier publications; original data or images not available; concerns about the images.

A GST-overlay assay was performed to determine whether the interactions between p53 and ZASP6, ZASP6-PDZ or ZASP6-ZM1 were direct or indirect (Figure 5C). Since recombinant proteins were expressed in bacteria and purified before use, there were no intermediary proteins available to mediate the interactions. In this experiment His-p53 recombinant protein was separated by SDS-PAGE and transferred to membranes. Strips were incubated with GST-ZASP6, GST-PDZ, GST-ZM1 or GST, and then probed with anti-GST polyclonal antibody. In the lower panel the second membrane was probed with an anti-histidine antibody, demonstrating that the same amount of His-p53 protein was loaded. Specific bands were detected indicating a direct interaction of p53 with full-length ZASP6 and ZASP6-PDZ, while no binding was observed between p53 and the ZASP6 ZM1 region (Figure 5C). The upper band detected in all of the blots is probably a non-specific bacterial contaminant from the His-p53 preparation that can be detected by anti-GST antibody.

Therefore only the interaction between the PDZ domain and p53 is direct, whereas the ZM1-p53 interaction probably needs another protein or proteins to act as intermediaries in the interaction. Requirement for post-translational modification (such as phosphorylation) of ZASP or p53 cannot be excluded.

### ZASP6, Ankrd2 and p53 form a Triple Complex

Ankrd2 is able to interact with p53 [42] and from the experimental results presented in this paper ZASP can bind both Ankrd2 and p53. Can these three proteins form a triple complex and, if so, what is the functional role of this triple complex? H1299 cells were used to express HA-ZASP6, GFP-p53 and cMyc-Ankrd2 proteins. Lysates from transfected cells were immunoprecipitated with immobilized anti-cMyc antibody and subsequently the immunocomplexes were probed with an anti-GFP HRP conjugated antibody (Figure 6A, row 1) and anti-ZASP antibody (Figure 6A, row 2). As controls the non-immunoprecipitated lysates were probed with anti-ZASP, anti-Ankrd2 and anti-GFP antibodies. The results of the Co-IP experiment demonstrated that Ankrd2 and ZASP6 were able to bind p53 independently of each other. Moreover, a triple complex was formed when the three recombinant proteins were over expressed (Figure 6A).

The article "ZASP Interacts with the Mechanosensing Protein Ankrd2 and p53 in the Signalling Network of Striated Muscle" was retracted in 2024. Reasons: duplicated images; overlap with earlier publications; original data or images not available; concerns about the images.

**Figure 6:** ZASP6, Ankrd2 and p53 are able to form a triple complex. (**A**) H1299 cells (p53−/−) were transfected with pcDNA3-HA-ZASP6, pcDNA3-p53 and pCMV3B-Ankrd2 as indicated. Transfected cell lysates were used for immunoprecipitation with anti-cMyc antibody. The top two panels represent the immuno-complexes separated by SDS-PAGE and blotted either with anti-GFP conjugated with HRP or anti-ZASP antibodies. Third, fourth and fifth panels represent Western blots of the extracts of transfected cells probed with anti-ZASP, anti-Ankrd2 and anti-GFP antibodies. The membrane where p53 was detected with anti-GFP antibody was stripped and reprobed with a mixture of anti SUMO-1 and anti-SUMO-2/3 antibodies (bottom panel). **B)** Co-IPs performed using lysates from H1299 cells transfected with pCMV2B-PDZ, pCMV3B-Ankrd2 and pEGFP-p53 as indicated. After immunoprecipitation with an anti-FLAG monoclonal antibody, SDS-PAGE and blotting, the membranes were probed with anti-Ankrd2 (first panel) or anti-p53 (second panel) antibodies. As controls, cell lysates were probed with anti-FLAG, anti-Ankrd2 and anti-p53 antibodies (respectively, third, fourth and fifth panels). **C)** *In vivo* interaction between ZM1, Ankrd2 and p53 was tested by co-immunoprecipitation of Ankrd2 and p53 with immunoprecipitated FLAG-ZM1 from lysates of the transfected H1299 cells using anti-FLAG antibody. Immuno-complexes were separated by SDS-PAGE, blotted and then probed with anti-Ankrd2 (first panel) and anti-GFP antibody conjugated with HPR (second panel). Expression levels of tested proteins were evaluated by Western blot, with anti-FLAG, anti-Ankrd2 and anti-GFP antibodies (respectively, third, fourth and fifth panel). **D)** GST overlay assay was performed by separating 4 μg of His-p53 by SDS-PAGE and blotting onto membranes. Strips were incubated with the same amounts (4 μg) of GST-PDZ, GST-Ankrd2, GST-ZASP6 and GST alone as indicated and probed in parallel with anti-GST (left panel), anti-Ankrd2 (middle panel) and anti-ZASP (right panel). The lower panel shows a Western blot of the cell lysates probed with an anti-Histidine monoclonal antibody to ensure that equal amounts of His-p53 recombinant protein was used.

The article "ZASP Interacts with the Mechanosensing Protein Ankrd2 and p53 in the Signalling Network of Striated Muscle" was retracted in 2024. Reasons: duplicated images; overlap with earlier publications; original data or images not available; concerns about the images.

It is interesting to note that several forms of p53, with different gel mobility, were present in cells co-expressing GFP-p53, ZASP6 and Ankrd2. The tumor suppressor p53 protein is extensively regulated by post-translational modification [56], including SUMOylation which is covalent attachment of small ubiquitin-related modifier (SUMO) to the protein target. The apparent molecular weight of the immunoprecipitated p53 would be consistent with the addition of one or two SUMO molecules to one GFP-p53 molecule. Therefore the same membrane was stripped and reprobed with a mix of SUMO-1 and SUMO-2/3 polyclonal antibodies. Only the two upper bands could still be detected but not the lower band of unmodified p53. Therefore these higher p53 forms that were detected by anti-SUMO antibodies (Figure 6A, last row) are SUMOylated forms of p53. It should be noted that SUMOylated p53 is only detected when p53 is co-expressed with Ankrd2 and ZASP together, not when p53 is co-expressed with either ZASP or Ankrd2 alone. This suggests that formation of the triple complex is possibly facilitated or enabled by SUMOylation of p53 (Figure 6A).

### ZASP6 PDZ Domain and Ankrd2 Interact Independently from p53

Since ZASP6, Ankrd2 and p53 form a triple complex, it was important to know if either the ZASP6 PDZ domain or the ZM1 region (protein without the PDZ domain) on their own are sufficient to interact in this triple complex.

Co-IPs were performed using lysates from H1299 (p53^−/−^) cells transiently transfected with different combinations of FLAG-PDZ, cMyc-Ankrd2 plus EGPF-p53 plasmids (Figure 6B). Transfected cell lysates were immunoprecipitated with anti-FLAG antibody and subjected to Western blotting. The presence of a triple complex was detected using anti-Ankrd2 and anti-p53 antibodies. It has already been demonstrated that the ZASP6 PDZ domain is able to bind Ankrd2 (Figure 2B) and p53 (Figure 5A). Here it can be seen that the presence of p53 did not impair this binding, hence we can deduce that not only do PDZ-ZASP6, Ankrd2 and p53 interact with each other (Figure 6B) but that this interaction was p53 independent, suggesting that there is no competition between PDZ-ZASP6 and p53 for the same binding site on Ankrd2.

### The Interaction of ZASP6-ZM1 and Ankrd2 is Blocked by p53

The ZASP6 ZM1 is able to bind Ankrd2 (Figure 2C) and p53 (Figure 5B) however the binding with p53 would seem to require an intermediary protein or proteins. Therefore it was interesting to see if it could form a triple complex with Ankrd2 and p53. To determine this, a Co-IP experiment was performed, H1299 cells were transfected with FLAG-ZM1, cMyc-Ankrd2 and EGFP-p53, individually or in combination, as indicated (Figure 6C). Lysates were immunoprecipitated with anti-FLAG antibody. Co-immunoprecipitated Ankrd2 and p53 were detected with anti-Ankrd2 and anti-GFP antibodies. An interaction between ZM1 and Ankrd2 was confirmed in the absence of p53. However the binding between the ZM1 and Ankrd2 was impaired when p53 was expressed in the cells, but binding between ZM1 and p53 occurred (Figure 6C). These data suggest a competition between proteins for a binding site. Whether p53 competes by blocking the binding site on Ankrd2 for the ZM1 or *vice versa* is not known, however it is clear that the interaction between the ZM1 and Ankrd2 is affected by the presence of p53.

The article "ZASP Interacts with the Mechanosensing Protein Ankrd2 and p53 in the Signalling Network of Striated Muscle" was retracted in 2024. Reasons: duplicated images; overlap with earlier publications; original data or images not available; concerns about the images.

Finally, to determine whether the interactions between the p53, Ankrd2 and ZASP6-PDZ or full length ZASP6 are direct rather than indirect an *in vitro* GST-overlay assay was performed. His-p53 recombinant protein detected by anti-Histidine antibody was used as loading control. The strips of the membrane were overlaid with the appropriate GST proteins; GST-PDZ plus GST-Ankrd2, GST-ZASP6 plus GST-Ankrd2 or as a control GST protein alone (Figure 6D). The detection was performed with anti-GST, anti-Ankrd2 and anti-ZASP antibodies. A series of specific bands were detected indicating that p53 bound directly to the complex of ZASP6-PDZ and Ankrd2, as well as the complex with ZASP6 full-length and Ankrd2. Therefore ZASP6 or ZASP6-PDZ, Ankrd2 and p53 can form a triple complex. It is probable that ZASP6 binds Ankrd2 in the presence of p53 via its PDZ region rather than the ZM1 region since this region is not able to bind Ankrd2 in the presence of p53.

### Localization of ZASP, Ankrd2 and p53

If interactions actually occur between these proteins they should at least be in the same vicinity within the cell. Immunofluorescence experiments were done to determine the localization of Ankrd2, ZASP and p53 in H1299 cells which do not express endogenous p53. They were co-transfected with the three constructs (pEGFP-ZASP6, pCMV-cMyc-Ankrd2 and pcDNA3-p53) separately, or in combination as shown in Figure S4. Indirect immunofluorescence was performed to analyze the pattern of fluorescence of each construct separately (Figure S4A). As expected, EGFP-ZASP6 was expressed in the cytoplasm, while Ankrd2 localized diffusely in both the nuclei and cytoplasm, defining the perinuclear boundary. p53 was confined to the nuclei (excluding nucleoli) however a small percentage also showed cytoplasmic fluorescence.

When H1299 cells co-expressed EGFP-ZASP6 and cMyc-Ankrd2 (Figure S4B) both retained same pattern as when transfected singly. In contrast to what was previously seen in cells transfected only with pcDNA3-p53, the p53 fluorescence was found exclusively in the nuclei (excluding nucleoli) but no additional cytoplasmic fluorescence was observed in the cells co-expressing ZASP6 and p53, while ZASP6 did not change its cytoplasmic pattern of localization (Figure S4B). When p53 is over-expressed in the cells together with Ankrd2, it retained exclusive nuclear localization, while the Ankrd2 appeared to be more highly expressed in the nucleus of the cell, although it was still present in the cytoplasm. Finally, the three proteins were over-expressed (Figure S4C) and the previously observed pattern was confirmed: ZASP6 localized in the cytoplasm, p53 appeared totally nuclear (excluding nucleoli) while Ankrd2 modified its pattern becoming more nuclear (although still diffused in the cytoplasm). Together, these data show that the expression of p53 in H1299 cells, which lack endogenous p53, may induce a nuclear accumulation of Ankrd2; however this does not affect the localization of ZASP6.

The article "ZASP Interacts with the Mechanosensing Protein Ankrd2 and p53 in the Signalling Network of Striated Muscle" was retracted in 2024. Reasons: duplicated images; overlap with earlier publications; original data or images not available; concerns about the images.

### The ZASP6-Ankrd2-p53 Triple Complex Affects p53-dependent Transactivation

It is known that p53 has a propensity to form complexes with other proteins, and that these p53-binding proteins seem to be important in determining whether p53 induces cell cycle arrest or apoptosis [57]. Dual luciferase assays were performed to determine whether the complex formed by ZASP6, Ankrd2 and p53 had any functional consequences on the p53 responsive promoters, MDM2 and BAX promoters. The *BAX* gene is involved in p53-mediated apoptosis and promotes cell death [58]. SaOs2 cells (null for p53), were co-transfected with the BAX promoter-LUC or the MDM2 promoter-LUC as well as the Renilla luciferase reporter gene and expression vectors for p53, ZASP6 and Ankrd2. Firefly luciferase activity was normalized to that of Renilla luciferase and presented as fold change relative to their activity when p53 alone was expressed (Figure 7). The co-expression of wild type p53 with Ankrd2 leads to an enhancement of p53-mediated transactivation of the both the BAX (Figure 7A) and MDM2 (Figure 7B) promoters. However ZASP6 co-expression led to a downregulation of p53 mediated transactivation of both the BAX (Figure 7A) and MDM2 (Figure 7B) promoters in the absence or presence of Ankrd2. This down-regulation was more pronounced for the BAX promoter. These results suggest that while Ankrd2 might act as an enhancer of p53 activity, ZASP6 appears to act as a negative regulator of p53 transcriptional activation both in the presence and absence of Ankrd2.

**Figure 7:** The effect of co-expression of ZASP6 and Ankrd2 on p53 transactivation of BAX and MDM2 promoters. Expression vectors for p53, ZASP6 and Ankrd2 were transiently transfected into SaOs2 cells along with a vector containing the Renilla luciferase reporter gene and (**A**) the BAX promoter-LUC or (**B**) the MDM2 promoter-LUC as indicated in the figure. The cells were lysed 16 h after transfection and luciferase activity was measured. Firefly luciferase activity was normalized to that of Renilla luciferase and presented as fold change relative to the activity when p53 alone was expressed. The plotted results were representative of three independent experiments performed in triplicate. Data were presented as means ± standard error of the mean. The Students t-test was done to determine the statistical significance, asterisks above the columns correspond to * p<0.05, **p<0.005.

The article "ZASP Interacts with the Mechanosensing Protein Ankrd2 and p53 in the Signalling Network of Striated Muscle" was retracted in 2024. Reasons: duplicated images; overlap with earlier publications; original data or images not available; concerns about the images.

## Discussion

The human ZASP protein has several isoforms due to alternative splicing. In order to harmonize the data from different sources we compiled a table (Table 1) cross-referencing the original nomenclature that hopefully will facilitate information retrieval. We also report a new isoform, ZASP8 which corresponds to Cypher 3c (Table S1). It should be noted that some of the eight isoforms are poorly expressed and ZASP3 may not exist. The functional significance of these isoforms is largely unknown however they are presumed to have different functions depending on their domain arrangements.

In contrast to the expression pattern seen in mouse where the isoforms that contain exon 6 are only expressed in skeletal muscle [18], in human these isoforms are expressed well in both skeletal and cardiac muscle [17] which was confirmed by the RNAseq data (Table 2). In fact, mutations in exon 6 have been detected in human heart associated with DCM [17]. The murine isoforms with exon 4 are expressed only in heart [18] whereas in human they are expressed in heart but also in skeletal muscle, albeit at a much lower level (Table 2). It is interesting that the human ZASP isoforms have a pattern of expression that correlates with the exon encoding the ZM-motif. ZASP2 and ZASP6 that have their ZM domain encoded by exon 6 are expressed well in both skeletal and heart muscle whereas ZASP1, ZASP5 and ZASP8 that have the ZM-motif encoded by exon 4 are expressed better in heart. The poorly expressed isoforms are those with two ZM-motifs (ZASP4 and ZASP7).

The RNA seq results can be partially corroborated by the expression profile of ZASP in human cardiac muscle that Leung et al [59] obtained during their identification of ZASP as the major O-linked β-N-acetylglucosamine substituted protein in human heart myofibrils. They were able to detect seven ZASP bands however they were only designated according to descending MW. From RNAseq data (Table 2) we detect three long isoforms (ZASP1, ZASP2 and ZASP8) and two short isoforms (ZASP5 and ZASP6) present in human heart. Unfortunately, a comparison between the isoforms designated ZASP1-7 in the Leung paper with those in Table 1 in this paper, is not possible due to the discrepancies in MWs and the possibility that some bands are products of protein cleavage [59].

The article "ZASP Interacts with the Mechanosensing Protein Ankrd2 and p53 in the Signalling Network of Striated Muscle" was retracted in 2024. Reasons: duplicated images; overlap with earlier publications; original data or images not available; concerns about the images.

As a premise to the discussion on ZASP protein dynamics, protein interaction experiments and reporter assays it should be noted that all of these experiments were done with over-expressed recombinant proteins in cultured cells that do not necessarily reflect the physiological conditions of endogenous proteins in muscle tissue, thus the information obtained, although valuable, is indirect.

Four human ZASP isoforms, two short ZASP5 and ZASP6 and two long ZASP1 and ZASP8 were studied. However, on studying their dynamic properties *in vivo* by FRAP, notable differences in their mobility were detected indicating that some forms were possibly involved in stable complexes. The ZASP6 isoform had the lowest percentage of mobile fraction (70%) but showed the highest K value (Table S4), reflecting high specificity of the binding that taken together with the low constant of dissociation value (Koff) indicates that this isoform is involved in stable and long lasting binding interactions. Moreover, the low kinetics of the curve (Figure 1A), indicate that the protein could be involved in an interaction of long duration with unknown binding partners or cytoskeletal structures [60].

ZASP8 shows intermediate kinetics typical of a protein involved in short transient bindings, while proteins ZASP1 and ZASP5 behave like monomeric proteins that are not or only very transiently involved in binding/unbinding interactions. ZASP1 and ZASP8 display different probabilities to undergo binding despite similar time of being in a bound state. A possible explanation could be that as only ZASP8 has exon 10, this exon may code for a region that binds one or more proteins interacting with ZASP, such as phosphoglucomutase1 [31]. Our results indicate that isoform dynamics did not seem to depend on molecular mass, nor the presence or absence of LIM domains but appear to be correlated to the difference in ZM-motif.

Can single point mutations perturb the dynamic properties of protein interactions? To answer this question we studied the interaction dynamics of some disease associated mutants of ZASP6 and ZASP1 by FRAP experiments (Figure 1B and 1C, Tables S4 and S5). Our results demonstrated that point mutations in exon 6, and especially within the ZM-motif, considerably modified the affinity of the mutated ZASP protein to interact with its binding partner(s) and also the selectivity of the binding decreases with respect to the ZASP6 wt protein. The pA165V mutant was particularly interesting as it has the highest Koff value and despite its ability to bind more frequently with respect to the other mutants, its binding time was the shortest. These data would suggest that this mutant is involved in transient bindings that are predominantly non-specific. On the basis of the FRAP data ZASP6 mutants did not totally lose their ability to bind, the interactions become more transient, unstable and non-specific depending on how close the mutation is to the core of the ZM-motif domain. In the case of the ZASP1 mutation pS189L, there is a decrease in the mobile fraction and the Koff value compared to the wt ZASP1, indicating that it has a lower ability to dissociate and its binding is more stable and specific, therefore it is probably bound to a fixed structure or confined in a cell compartment (Figure 1C, Table S5). Recently, ZASP1 has been reported as a protein kinase A (PKA) anchoring protein [61]. The same mutation S189L did not change the interaction between ZASP1 and PKA although from the FRAP results it would be expected to bind PKA stronger than ZASP1. The discrepancy between these two data sets could be explained by different experimental settings since FRAP reflects an *in vivo* situation, with all sarcomeric proteins present, while Lin and co-authors used ZASP1 and PKA protein fragments over-expressed in non-muscle cells [61]. In conclusion, our results further support already demonstrated importance of the integrity of the ZM-motif for both binding specificity and stability [24], [25]. Mutations in the ZM-motif of ZASP6 reduced the binding affinity for its partners whereas the mutation ZASP1_S189L had the opposite effect. However the possible partners involved in these interactions are unknown. The data obtained from the FRAP experiments would appear to validate the initial hypothesis of the importance of the ZM-motif and provide evidence of how an impairment of this binding site totally modifies the dynamics and protein-protein interaction of the ZASP protein. As mentioned previously these experiments are performed in myoblasts that have not yet developed Z-bodies or Z-lines so they only provide indirect evidence as to what might happen at the Z-line.

The article "ZASP Interacts with the Mechanosensing Protein Ankrd2 and p53 in the Signalling Network of Striated Muscle" was retracted in 2024. Reasons: duplicated images; overlap with earlier publications; original data or images not available; concerns about the images.

Many Z-line proteins are known to have more than one binding partner, interacting directly or indirectly, to form part of a complex network of proteins [39], [62]. Here we identified two novel ZASP interacting proteins, namely Ankrd2 and p53. Ankrd2 is expressed in the nucleus of myoblasts, however upon their differentiation into myotubes it is expressed in the cytoplasm [42], [45]. Overexpression of Ankrd2 inhibits differentiation [63], [64]. Further indication of the importance of Ankrd2 was the finding that oxidative stress caused by hydrogen peroxide activated the Akt2 mediated phosphorylation of Ankrd2 (Ser-99) [45]. Moreover, expression of a phosphorylation defective mutant (S99A) resulted in faster differentiation. The assumption is that under stress conditions Akt-dependent phosphorylation is involved in the negative regulation of myogenesis [45]. Ankrd2 can bind directly to the ZASP6 PDZ region as well as a site or sites in the ZM1 region (Figure 2), the site on Ankrd2 involved in this binding is the ankyrin repeat region (Figure 3). Apart from titin and telethonin [41], [65], ZASP is another Z-line protein which interacts with Ankrd2 via its ankyrin repeats. In fact, we had proposed that ankyrin repeats are sufficient to enable participation of Ankrd2 in building sarcomeric multiprotein complexes.

All of the mutants studied were able to bind both alpha-actinin2 (Figure 4A) and Ankrd2 (Figure 4B) with the exception of the mutants in the ZM-motif ZASP6_A165V and ZASP6_A171T (Figure 4B) that showed no binding to Ankrd2 but weak binding to alpha-actinin2, possibly due to residual binding to their PDZ domain.

p53 is a key player in signalling pathways for the regulation of cell growth and apoptosis induced by stress [66], [67]. In unstressed cells p53 protein levels are kept low by degradation via the action of MDM2 [68]. However if the auto-inhibitory feedback loop is broken due to p53 being unable to transactivate the MDM2 promoter then p53 is stabilized and not targeted for degradation [69]. Mild stress results in cell cycle arrest via the upregulation of p21, a cyclin-dependent kinase inhibitor [70]. Severe or prolonged stress leads to apoptosis via p53 activation of *BAX5* and *PUMA* [71] as well as by repression of anti-apoptotic [72] and cell cycle [73] genes. Recently there have been reports of p53 upregulation in muscle being linked to muscle atrophy in Huntington’s disease [74] and LGMD2C [75]. Another case of p53 being associated with muscle weakness is ageing, in which there is a notable loss of muscle mass and an increase in adipose tissue resulting in a decline in skeletal muscle [76]. Elevated levels of p53 in human DCM were associated with a dysregulation of the ubiquitin-proteasome system which regulates p53 stability [77]. High levels of p53 have also been associated with caspase activation in HCM in response to pressure overload, as well as with higher phosphorylation and nuclear localization of p53 protein in Duchenne muscular dystrophy [78], [79]. Previously we showed that Ankrd2 interacted with p53 enhancing its function as a transactivator of the p21 promoter [41], [42]. Here we show interaction between ZASP and p53, both ZASP full length and its PDZ domain alone can bind directly to p53 (Figures 5A and 5C). However the ZM1 region can only bind indirectly to p53 (Figures 5B and 5C) therefore it may require another protein or proteins to act as intermediary in binding p53.

The article "ZASP Interacts with the Mechanosensing Protein Ankrd2 and p53 in the Signalling Network of Striated Muscle" was retracted in 2024. Reasons: duplicated images; overlap with earlier publications; original data or images not available; concerns about the images.

Since Ankrd2, ZASP and p53 interact with each other, we speculated that they could form a complex. The result of this study provides the first evidence that ZASP6, Ankrd2 and p53 are able to form a trimeric complex (Figure 6). The PDZ domain on its own was sufficient to interact with Ankrd2 and p53 in the triple complex, indicating that this interaction is p53 independent, which suggests that there was no competition between PDZ-ZASP and p53 for the same binding site on Ankrd2. Indeed the presence of p53 appears to amplify the intensity of the detected band, it is possible that it could stabilise the binding between the ZASP6 PDZ and Ankrd2. However, unlike the result with the ZASP PDZ domain, the interaction between ZM1 and Ankrd2 did not occur if p53 was over-expressed in the cells suggesting a competition between these proteins for the same binding site. Whether p53 competes by blocking the binding site on Ankrd2 for ZM1 or vice versa is not known. Although the triple complex can be formed *in vitro* more experimental evidence is needed to confirm its existence *in vivo*. It should be noted from the literature [80] that under certain circumstances, such as stress conditions, p53 can be found in the cytoplasm. It is possible that interaction with ZASP could sequester p53 in the cytoplasm, however this is purely speculative and we have no proof that this occurs *in vivo.*

From our results we can deduce that the ZASP6 PDZ domain binds to Ankrd2 via its ankyrin repeat region whereas the ZASP6 ZM1 could have the same binding site as p53 on Ankrd2. We previously showed that, in addition to ankyrin repeats, N-terminal region of Ankrd2 is required for interaction with p53 as well as transcription factors YB-1 and PML [42]. We can speculate that the ankyrin repeats are able to accommodate more than one binding partner and that binding specificity is achieved by concurrent interaction with the N terminal region that is proximal to ankyrin repeats.

An intriguing finding is that p53 is modified by SUMO when present in the triple complex (Figure 6). This endogenous poly-SUMOylation of p53 was detectable only in the presence of full-length ZASP6. If the ZASP6 PDZ domain or ZM1 region were co-expressed with Ankrd2 and p53, SUMO modified p53 was never detected in the complex. However which SUMO family member is involved in the modification of p53 in the trimeric complex is not known since the mixture of antibodies specific for SUMO1 and SUMO2/3 was used. p53 is SUMOylated at a single site K386 [81] by SUMO-1 [82] and SUMO-2/3 [83]. Modification of p53 via SUMO-2/3 or SUMO-1 can have different consequences. SUMO-1 modification of p53 results in nuclear export of p53 [84], however that does not appear to happen when p53 is modified by SUMO-2/3 [85].

The article "ZASP Interacts with the Mechanosensing Protein Ankrd2 and p53 in the Signalling Network of Striated Muscle" was retracted in 2024. Reasons: duplicated images; overlap with earlier publications; original data or images not available; concerns about the images.

The SUMOylation of p53 seen in the presence of the triple complex could possibly result in a modification of the action of p53 probably by facilitating its cytoplasmic export whereas a block of the SUMOylation could probably result in p53 retention in the nucleus. The ZASP6 ZM-motif mutants unable to bind Ankrd2 (ZASP6_A165V and ZASP6_A171T) could disrupt the formation of the triple complex and therefore SUMOylation of p53 by interfering with the binding of p53 and Ankrd2. Another possibility is that SUMOylation of p53 is needed as an additional platform to enable interaction with full length proteins, while unmodified p53 is able to accommodate Ankrd2 and ZASP deletants (PDZ or ZM1). Attachment of SUMO facilitates protein–protein interactions, either by creating new interaction surfaces or by indirectly affecting the conformation of the modified target, thereby facilitating the assembly of multi-protein complexes, the recruitment of regulatory factors to the site of modification or the sequestration of the target into different subcellular compartments [86].

Promoter assays were performed to determine if the interaction of ZASP6 with Ankrd2 and p53 could have any functional consequence on the ability of p53 to transactivate responsive promoters (Figure 7). Two different promoters were used in luciferase assays to test this hypothesis: the BAX promoter that regulates the expression of Bax (Bcl2-associated X protein) and the MDM2 promoter that regulates the expression of the Mdm2 protein, a potent inhibitor of p53 transcriptional activation [87]. Ankrd2 enhanced the p53-mediated activation of both the BAX and MDM2 promoters, while ZASP6 acted as a negative regulator of p53 transcriptional activation both in the presence and absence of Ankrd2. Further experimental evidence is needed in order to elucidate the possible influence of ZASP and Ankrd2 on p53 function. The question is when and why ZASP acts to attenuate p53 transactivation and how Ankrd2 is involved. Since.

ZASP can interact with p53 preventing it to activate p53 responsive genes, ZASP can also be involved in mechanoptosis, similarly to what is proposed for telethonin. Mechanoptosis is defined as a type of apoptosis induced via mechanical stress [62]. The increase in sarcomere activity is translated into pro-survival signals by sequestering p53 in cytoplasm. Telethonin interferes with p53 in nucleus, but we can propose an additional mechanism of cytoplasmic sequestration of p53 when muscle cells are challenged and sarcomeroptosis is activated. Ankrd2 could also be sequestered thus preventing the activation of p53 in nucleus.

The article "ZASP Interacts with the Mechanosensing Protein Ankrd2 and p53 in the Signalling Network of Striated Muscle" was retracted in 2024. Reasons: duplicated images; overlap with earlier publications; original data or images not available; concerns about the images.

The study of Lin and colleagues [61] on PKA and ZASP directly connects Cypher/ZASP to the signal transduction pathways via participation in signaling that regulates the phosphorylation of some proteins, including the L-type Ca+ channel (LTCC) and Cypher/ZASP itself. In cardiomyocytes they show that not only does Cypher/ZASP interact with the regulatory subunit of PKA acting as physical anchor but that it was also phosphorylated by it at Ser265 and Ser296. Also the Cypher/ZASP PDZ domain enhanced PKA phosphorylation of LTCC protein by binding via its C-terminal PDZ binding motif. Another interesting fact was that they showed Cypher/ZASP binding to calcineurin, a serine/threonine phosphatase of the LTCC. These and our findings connecting ZASP to the p53 pathway are in line with the concept that in cardiac Z-lines ZASP not only has a structural function but also a role in signaling [39]. Other intriguing information in this regard is that ZASP can bind proteins of the FATZ/calsarcin/myozenin family (27, 28) that in turn are known to bind and regulate calcineurin [88].

In conclusion, here we describe the expression pattern and dynamic properties of ZASP isoforms and disease associated mutants of ZASP. Ankrd2 and p53 were identified as new binding partners of ZASP. Moreover, these three proteins are able to form a trimeric complex, potentially involved in signaling, regulation of gene expression and muscle differentiation. Endogenous poly-SUMOylation of p53 occurred but only in the triple complex in the presence of ZASP6. ZASP6 was shown to be a negative regulator of p53, at least for transactivation of the p53-responsive promoters MDM2 and BAX. On studying disease associated mutations in ZASP6 we found that two ZM-motif mutants, A165V and A171T, were not able to bind Ankrd2. This is the first indication of how mutant ZASP protein can differ from wild type and is particularly important since the A165V mutation is responsible for a well characterized autosomal dominant distal myopathy, zaspopathy. Although still unknown, the mechanism by which this mutant causes MFM may involve disruption of the heterotrimeric complex by blocking p53 SUMOylation.

The article "ZASP Interacts with the Mechanosensing Protein Ankrd2 and p53 in the Signalling Network of Striated Muscle" was retracted in 2024. Reasons: duplicated images; overlap with earlier publications; original data or images not available; concerns about the images.

## Materials and Methods

### Antibodies

The following antibodies were produced by us: anti-Ankrd2 mouse monoclonal antibody (clone 2F10), made using the C-terminal region of Ankrd2 (aa 324–360); anti-FL Ankrd2 rabbit polyclonal antibody, raised in rabbits against the His tagged human Ankrd2 protein (aa 32–360); anti-FL Ankrd2 mouse polyclonal antibody, raised in mice against His-tagged human Ankrd2 protein (32–360 aa) [41], [42], [44]. Anti-ZASP polyclonal antibody was produced in mice against His-tagged human ZASP6 (1–283 aa) [9]. Rabbits and BALBc mice were purchased from Charles River Laboratories Italia Srl and maintained under controlled environmental conditions. Animal care and treatment was in compliance with national and international laws and policies (European Economic Community Council Directive 86/609, OJL 358, December 12, 1987, and current Italian law, decree 116/92). The commercial antibodies were used according to the manufacturer’s protocol.

### Cell Culture, Transfections and Preparation of Protein Extracts

COS-7 (CRL-1651), SaOs2 (HTB-85), H1299 (CRL-5803) and C2C12 (CRL1772) cells were obtained from the ATCC (Manassas, VA, USA). COS-7 cells and C2C12 mouse myoblasts were maintained in DMEM containing 10% (v/v) fetal calf serum (FCS) and gentamycin (50 μg/mL) whereas SaOs2 cells were grown in the same medium but with 20% FCS. For FRAP experiments C2C12 cells were maintained in medium containing DMEM without phenol red. Primary human myoblasts CHQ5B cells were obtained and grown as described previously [9].

### ZASP Constructs

The full-length ZASP6 human cDNA (1–849 bp) [9] was cloned into the following expression vectors: pQE30 (Qiagen); pGEX-6PH-3, a modified form of the pGEX-6P-3 vector (GE Healthcare); pCMV-2B (Stratagene); pcDNA3-HA, a modified form of the pcDNA3 vector (Invitrogen); pEGFP-C1 (CLONTECH), respectively, expressing His, GST, FLAG, HA, and GFP tagged ZASP6 recombinant proteins. Both the PDZ (1–255 bp) and ZM1 (258–849 bp) regions of human ZASP6 isoform were amplified by PCR using the ZASP6-pCMV2B construct as a template and then cloned into the following vectors pQE30 (Qiagen), a modified version of pGEX-6-P3 (GE Healthcare) and pEGFP-C1 (CLONTECH). The ZM1 region is basically the full length ZASP6 without the PDZ region and includes the ZM-motif. The full-length ZASP1, ZASP5 and ZASP8 isoforms were amplified by PCR and cloned into the pEGFP-C1 vector (CLONTECH) that expresses a N-terminal GFP tagged recombinant protein.

### Site-directed Mutagenesis

The full-length ZASP1-pEGFP-C1 and ZASP6-pEGFP-C1 constructs were subjected to site directed mutagenesis using a QuikChange II XL Site Directed Mutagenesis Kit (Agilent) according to the manufactuer’s protocol. The mutants produced (ZASP1_S189L, ZASP6_A171T, ZASP6_A147T, ZASP6_A165V) and their specific primers are listed in Table S6. The mutated cDNAs were cloned directly into the *Bam*HI-*Hind*III restriction sites in the following vectors: pCMV-2B, pCMV-3B and pEGFP-C1, respectively, expressing FLAG, cMyc and GFP tagged recombinant proteins.

The article "ZASP Interacts with the Mechanosensing Protein Ankrd2 and p53 in the Signalling Network of Striated Muscle" was retracted in 2024. Reasons: duplicated images; overlap with earlier publications; original data or images not available; concerns about the images.

### Ankrd2 and p53 Constructs

Human Ankrd2 cDNA (96–1,080 bp) was cloned into pcDNA3.1 (Invitrogen) and the following expression vectors: pQE30 (Qiagen), pCMV-2B and pCMV-3B (Stratagene) as well as a modified version of pGEX-6-P3 (GE Healthcare) expressing respectively His, FLAG, cMyc and GST tagged recombinant proteins. The cDNA’s corresponding to different fragments of the Ankrd2 gene (96–441 bp; 96–933 bp; 444–1,080 bp; 918–1,080 bp) were inserted into the pGEX-6P-3 vector. These cDNAs correspond to the following protein regions: N-terminus (N, 32–147 aa), N-terminus plus Ankyrin repeats (NA, 32–311 aa), C terminus plus Ankyrin repeats (CA, 148–360 aa) and C-terminus (C, 306–360 aa). The p53-pGEX-2T construct was kindly supplied by Dr. L. Banks (ICGEB, Trieste, Italy), the p53-pcDNA3 was kindly provided by Dr. G Del Sal (University of Trieste, Trieste, Italy). The cDNA of full length p53 was cloned into the pQE30 and pEGFP-C1 vectors expressing respectively, His and GFP tagged recombinant proteins.

### Quantitative Real-Time PCR (qPCR)

Total RNA quality was assessed using an Agilent 2100 bioanalyzer to obtain an accurate reading of the 18S and 28S peaks. Using the TaqMan chemistry, we designed probes and primers, which are available upon request, to quantify the expression levels of all known ZASP isoforms. qPCR was performed on the commercial human total RNA from either skeletal or cardiac muscle at the BCM Microarray Core (Baylor College, Houston, Texas) using the iCycler iQ Real-Time PCR Detection System (BioRad, Hercules, CA).

### Whole Transcriptome Library Preparation

Either poly (A) or total RNA was used for the RNA fragment library preparation. The RNA was digested by RNase III, the resulting fragments prepared using a Ribominus concentration module (Invitrogen) and its size was assessed using an Agilent Bioanalyzer. Depending on the sequencing platform either a SOLiD transcriptome multiplexing kit or an Ion Xpress RNA seq barcode kit were used to prepare “barcoded” libraries which enables sequencing of multiple transcriptome samples in a single multiplexed sequencing run. Ligated RNA was reverse transcribed and the resulting cDNA was purified and size selected using magnetic beads to obtain 100–200 nt cDNA. The size selected cDNA was then amplified using 5′ SOLiD and 3′ barcoded SOLiD primers. Each SOLiD barcoded 3′ primer contains the sequence required for SOLiD emulsion PCR, a unique 6 nucleotide barcode sequence, and an internal adaptor sequence necessary for sequencing the barcode. The amplified DNA was then purified and its quality was assessed using Agilent Bioanalyzer to ascertain that the DNA is 25–150 bps. Barcoded libraries were pooled prior to template bead preparation and emulsion PCR following the manufacturer’s protocol was performed. The samples were sequenced on either a SOLID or ION-Proton machine (Life Technology).

The article "ZASP Interacts with the Mechanosensing Protein Ankrd2 and p53 in the Signalling Network of Striated Muscle" was retracted in 2024. Reasons: duplicated images; overlap with earlier publications; original data or images not available; concerns about the images.

### RNAseq

SOLiD reads were mapped to the reference human genome (hg19) using PASS program, version 2.11 [89], the percentage identity was set to 90%, and one gap was allowed. The quality of the filtering parameters was set automatically by PASS. The spliced reads were identified using the procedure described in the PASS manual which can be found at the following link (http://pass.cribi.unipd.it). The Ion Proton reads were first cleaned by removing the adaptor sequence, using the program cutadapt [90] and then mapped using the program GSNAP [91] with default parameters except for the percentage identity that was set to 90%. Gene annotation (release 72) was downloaded from the ENSEMBL ftp site and isoform quantification was performed using Cufflinks software, version 2.1.1 [49]. Cufflinks was run using the bias correction option to improve the estimate of accuracy of transcript abundance [92]. The splicing site coverage analysis was performed using a home-made python script. Briefly, for each transcript model the script extracts the splicing site coordinates and the RNAseq spliced read coordinates were then used to verify and confirm each splicing site. Three different analyses were performed setting to, 1, 2 and 5, respectively, the minimum number of spliced reads to support a splice site. An isoform was considered to be expressed only if all its splicing sites were confirmed. The RNAseq data were based on three different biological replicates for adult skeletal muscle and two for adult cardiac muscle, while the results obtained for foetal cardiac and skeletal muscle were from only one RNAseq experiment.

### Immunofluorescence

Mouse myoblasts (C2C12) and a lung cancer cell line (H1299, p53^−/−^) were grown on collagen-coated (Rat Tail Collagen Type I, Becton Dickinson Labware) coverslips and transfected the next day. They were fixed with 3.5% formaldehyde, then treated with 0.1M Glycine and permeabilised by incubating in PBS/0.1% Triton X-100. Any non-specific binding was blocked with 1% BSA (Bovine Serum Albumin, SIGMA). All washing steps and antibody dilutions for these experiments were performed with PBS/0.1% BSA/0.05% Tween 20. The samples were incubated for 90 min with primary antibodies, washed and then stained with secondary antibodies. All commercial immunochemicals were diluted as recommended by the suppliers. The actin cytoskeleton (F-actin) was visualized with Rhodamine-Phalloidin (P1951 Sigma). The coverslips were mounted on slides with Vectashield (VECTOR Lab Inc, Burlington, USA) and examined by confocal microscopy performed with a Zeiss LSM 510 META Confocal Microscope (Carl Zeiss Microscopy, Jena, Germany), using a 100x oil immersion objective.

The article "ZASP Interacts with the Mechanosensing Protein Ankrd2 and p53 in the Signalling Network of Striated Muscle" was retracted in 2024. Reasons: duplicated images; overlap with earlier publications; original data or images not available; concerns about the images.

### Fluorescence Recovery after Photobleaching (FRAP)

Experiments were performed with the Zeiss LSM 510 META Confocal microscope (Carl Zeiss, Jena, Germany) using a 63 × oil immersion objective with an excitation wavelength of 488 nm (1.05% laser power) and a band-pass 505–530 nm emission filter from a 30.0mW Argon/2 laser operating at 75% laser power. C2C12 were plated on 35 mm glass bottom dishes coated with poly-d-lysine (MatTek Corporation) and transfected with 1.5 μg of DNA using FuGENE 6 (Roche, Basel, Switzerland) as directed by the manufacturer. FRAP recordings were performed 24 h post-transfection, under following conditions: resolution of 512×512 pixels, at maximum speed (one image every 983.04 ms) and zoom 2X. Bleaching was performed with a rectangle ROI (inside the cytoplasm of the cell) with the laser at 100% power. Post-bleach images were monitored at low laser intensity at 10 sec intervals. Data were analysed using MetaMorph software (Molecular Devices). Stacks of images in each time series were aligned and the average fluorescence intensity of the bleached cytoplasm, unbleached cytoplasm as a control and a background region, were recorded for each time point. For the data analysis, background was subtracted and fluorescence intensity was normalized as described by Phair and Misteli [53]. The fluorescence recovery curves were fitted with a reaction-diffusion model for rectangular roi (Table S5) [54] and the mobile fraction (MF), rates of binding and unbinding and half time recovery (t1/2), were obtained from the fit. The number of samples was 15–20 different cells for each FRAP analysis. Grouped data are presented as the mean ± standard deviation (SD).

### Transfection and Co-immunoprecipitation

Sub-confluent COS-7 cells and p53^−/−^ H1299 and SaOS-2 cells were transfected with the appropriate expression vectors using the FuGENE 6 reagent (Roche) as described in the manufacturer’s protocol. Lysates were made 48 hr after transfection, in E1A buffer (50 mM Hepes pH 7, 250 mM NaCl, 0.1% v/v NP40) supplemented with protease inhibitors (Complete-EDTA free, Roche). Samples were briefly sonicated and cleared by centrifugation. The protein concentration was determined using a Protein Assay (Biorad). Tagged proteins were immunoprecipitated from the extracts by specific antibodies for 2 hours at 4°C and protein A-Sepharose (GE Healthcare) for additional 1 hour. After five brief washings in binding buffer, proteins were eluted from the beads by boiling samples in DTT containing sample buffer and subjected to SDS-PAGE. The presence of specific proteins in immunocomplexes was determined by Western blotting. The antibodies used for immunoprecipitation were: anti-c-Myc clone 9E10 mouse monoclonal ascites fluid (M5546, Sigma), anti-HA (F-7) mouse monoclonal antibody (sc-7392, Santa Cruz Biotechnology, Inc.) and anti-p53 (DO-I) mouse monoclonal antibody, isotype IgG2a (Sc-126 Santa Cruz Biotechnology, Inc). Resin immobilized antibodies to cMyc and FLAG tags, EZviewTM Red Anti-cMyc Affinity Gel (E6654, Sigma) or EZview Red Anti-FLAG M2 Affinity Gel (F2426, Sigma), were also used.

The article "ZASP Interacts with the Mechanosensing Protein Ankrd2 and p53 in the Signalling Network of Striated Muscle" was retracted in 2024. Reasons: duplicated images; overlap with earlier publications; original data or images not available; concerns about the images.

### Western Blotting

Protein complexes, resolved by SDS PAGE, were transferred to PVDF membrane (Immobilon P, Millipore) as previously reported [42]. Following primary antibodies were used: anti-ZASP mouse polyclonal (1∶1000–1∶1500 dilution), anti-HA (F-7) mouse monoclonal (1∶300 dilution), anti-FLAG M2 monoclonal antibody (1∶300 dilution), anti-FLAG rabbit polyclonal (1∶500 dilution), anti-Ankrd2 mouse polyclonal (1∶800 dilution), anti-Ankrd2 mouse monoclonal (1∶200–1∶400 dilution), anti-c-Myc mouse monoclonal (1∶300 dilution), anti-p53 DO-1 mouse monoclonal (1∶500 dilution), anti-GFP rabbit polyclonal (1∶1000 dilution), anti-goat GFP HRP-conjugated (1∶1000 dilution), anti-6xHis mouse monoclonal (1∶2000 dilution) and anti-goat GST polyclonal (1∶5000 dilution). Anti-mouse and anti-rabbit antibodies conjugated with horseradish peroxidase (Sigma and Pierce, respectively) were used as the secondary antibodies. Proteins were visualized using the Enhanced Chemiluminescence Kit (ECL, GE Healthcare).

### GST-pull Down Assay

Equal amounts of GST fusion proteins bound to glutathione-Sepharose 4B matrix were incubated for two hours at 4°C with protein extract (300 μg) from transfected COS-7 cells. After washing, the samples and a control consisting of 20% of the total lysate used in each of the binding reactions were separated by SDS-PAGE, transferred to membrane and subjected to Western blot detection.

### GST-overlay Assay

Purified His-tagged proteins (4 μg) were subjected to SDS-PAGE and then blotted onto Immobilon-P membrane (Millipore). The membranes were blocked in 10% low fat milk in PBS with 0.05% Tween 20 to avoid non-specific interactions and then incubated either with purified GST fused recombinant proteins or GST alone (4 μg). After five washings the membranes were incubated with an antibody against GST (anti-GST goat polyclonal, GE Healthcare, 1∶1000 dilution) and anti-goat HRP conjugated antibody (Santa Cruz Biotechnology Inc., 1∶5000 dilution). The signals were developed using ECL (GE Healthcare).

The article "ZASP Interacts with the Mechanosensing Protein Ankrd2 and p53 in the Signalling Network of Striated Muscle" was retracted in 2024. Reasons: duplicated images; overlap with earlier publications; original data or images not available; concerns about the images.

### Reporter Gene Assay

The Dual-Luciferase Reporter Assay System (Promega) was used to carry out transactivation experiments using BAX and MDM2 promoters cloned upstream of the Firefly luciferase reporter gene. SaOs2 cells were grown for 24 h and then transiently co-transfected using Lipofectamine 2000 (Life Technologies) with reporter vectors (500 ng of BAX promoter-LUC or MDM2 promoter-LUC and 100 ng of Renilla luciferase reporter) and expression vectors for p53, ZASP6 and Ankrd2. The cells were lysed in Passive Lysis Buffer (Promega) 16 h after transfection and luciferase activity was measured using the Dual-Luciferase Assay System (Promega) and TD-20/20 Luminometer (Promega). Firefly luciferase activity was normalized to that of Renilla luciferase. Plotted results are representative of three independent experiments performed in triplicate. Data were presented as means ± standard error of the mean. The Students t-test was done to determine the statistical significance (the accepted level was p<0.05).

## Supporting Information

Figure S1 **qPCR of human ZASP isoforms.** Relative ZASP Isoform/GAPDH ratio was calculated using the Ct (threshold cycle) of the reference gene (GAPDH) versus the isoform target using quantitative (real-time) polymerase chain reaction (qPCR) to determine the level of expression of ZASP isoforms in adult human heart (H) and skeletal muscle (S). Group1, ZASP isoforms 2, 3 and 6; Group2, ZASP isoforms 1, 5 and 8, and Group3, ZASP isoforms 4 and 7.
(TIF)

Figure S2 **Localization of GFP-tagged ZASP isoforms in C2C12 cells.** Human GFP tagged ZASP isoforms: ZASP1, ZASP5, ZASP6, and ZASP8 were expressed in C2C12 cells. **A**) The actin was stained with rhodamine-phalloidin (red) and the localization of the GFP tagged ZASP isoforms (green) was noted to be along the actin cytoskeleton. **B)** Alpha-actinin2 was stained with monoclonal anti-actinin2 antibody and anti-mouse Texas Red (red). The ZASP isoforms were detected by their GFP tag (green). There was co-localization of the ZASP isoforms and alpha-actinin2. All the pictures were captured using a laser scanning Meta Confocal microscope (Zeiss) with 100x objective (Bar = 10 μm).
(TIF)

Figure S3 **FRAP experiments in murine myoblasts.** C2C12 cells were transfected with pEGFP constructs expressing GFP tagged human ZASP isoforms: GFP-ZASP1, GFP-ZASP5, GFP-ZASP6 and GFP-ZASP8. Images shown from left to right are pre-bleached, bleached and recovery after bleaching at different time points. All the pictures were captured using a laser scanning Meta Confocal microscope (Zeiss) with 63x objective (Bar = 5 μm).
(TIF)

Figure S4 **Localization and co-localization of GFP-ZASP6, cMyc-Ankrd2 and p53 in H1299 cells.** H1299 cells which do not express endogenous p53 were cultured and transfected with each of the three constructs (pEGFP-ZASP6, pCMV-cMyc-Ankrd2 and pcDNA3-p53) or in combination. **A)** single transfections; Ankrd2 was detected using a rabbit polyclonal antibody to human FL-Ankrd2 and anti-rabbit Texas red as the secondary antibody. p53 was detected with a mouse anti-p53 (DO-1) monoclonal antibody and anti-mouse Texas Red as the secondary antibody. **B)** double transfections; cells expressing GFP-ZASP and cMyc-Ankrd2 were probed with a rabbit polyclonal antibody to FL-Ankrd2 and anti-rabbit Alexa Fluor 633 as the secondary antibody. When co-expressing GFP-ZASP and p53, cells were probed with mouse anti-p53 (DO-1) and anti-mouse Texas Red as the secondary antibody. **C)** Indirect immunofluorescence performed on triple transfected cells using as primary antibodies, mouse monoclonal anti-p53 (DO-1) and a rabbit anti-FL-Ankrd2. The secondary antibodies used were anti-mouse Texas Red (red) and anti-rabbit Alexa Fluor 633 (blue). All the pictures were captured using a laser scanning Meta Confocal microscope (Zeiss) with 100x objective (Bar = 10 μm).
(TIF)

Table S1 **Comparison of Cypher and ZASP isoforms.**
(DOC)

Table S2 **Splicing site coverage analysis.**
(XLS)

Table S3 **Detailed RNAseq analysis data for human ZASP isoforms.**
(XLS)

Table S4 **FRAP data for ZASP isoforms and mutants.**
(DOC)

Table S5 **Detailed fit values for ZASP isoforms and mutants.**
(XLS)

Table S6 **Primers for site-directed mutagenesis for ZASP1 and ZASP6 mutants.**
(DOC)
